# Impact Analysis of Environmental Regulation and Improvement of Agricultural Economic Efficiency on Living Environment Based on Systematic GMM Model

**DOI:** 10.1155/2022/7674549

**Published:** 2022-07-09

**Authors:** Jiahui Zhu, Bin Zhou, Wenhan Li

**Affiliations:** ^1^Xi'an University of Science and Technology, Xi'An 710000, China; ^2^University of Surrey, Surrey, Guildford GU2 7XH, UK

## Abstract

The living environment is of vital importance to human beings and is also the basis for their survival and development. Along with the accumulation of people's production and living experience, people are seeking their own development while studying the living environment more deeply. In recent years, various regions and departments have conscientiously implemented the relevant decisions and deployments. They have promoted the construction of rural infrastructure and the equalisation of basic public services between urban and rural areas, so that the rural living environment can be gradually improved. The rapid development of urban-rural integration has brought great opportunities and challenges for rural development, making rural development issues increasingly complex and affecting the effectiveness of the construction of a new rural habitat. At the same time, the agricultural economy is the basis of national economic development, and the ecological environment provides a certain amount of material environment for the development of the agricultural economy. Therefore, research on the harmonious development of the agricultural economy and the ecological environment has always been a hot issue for the authorities concerned. After all, China's agricultural economic development mode is characterized by a rough-and-ready approach, and the agroecological environment continues to deteriorate, leaving the issue of sustainable agricultural development to be resolved. What is worse, in the practice of agricultural production, the related agricultural activities have brought serious pollution to the environment. Specifically, the carrying capacity of the agricultural ecological environment is declining, leading to an increasingly serious conflict between sustainable agricultural economic development and the construction of an environmentally friendly and resource-saving society. In China, although the industrialization process is accelerating, the agricultural population still accounts for a large proportion of the population. As people's living standards continue to improve, a favorable living environment has become an urgent need for farmers. As a result, strengthening the construction of rural infrastructure, improving rural living conditions, and improving rural environmental sanitation are important issues that need to be addressed urgently. Therefore, to further investigate the impact of environmental regulation and agricultural economic efficiency on the habitat, this study constructs a systematic GMM model using panel data for 30 provinces and regions in China from 2011 to 2021.

## 1. Introduction

Since the reform and opening-up, China's economic growth has been driven by a combination of internal and external factors, such as marketization, and it has moved from a rough and tumble stage of development to a modern and fine-grained transition stage. Accordingly, China's economic development has resulted in the upgrading of its agricultural industry. From Figure 1, it can be seen that the agriculture industry is the most important industry in China. As a basic industry for China's economic construction and development, agriculture should pay more attention to the coordinated and sustainable development of the agricultural economy and the agroecological environment to further consolidate the basic position of agriculture in the development of the national economy. Agriculture is a combination of natural and economic reproduction processes [1]. Changes in agricultural factors and technological conditions result in a differentiated distribution pattern of agricultural industries. As a result, it is the most correct choice in China's economic construction to adhere to the strategic policy of achieving high-quality agricultural development and improving the efficiency of the agricultural economy [2]. Also, the construction industry is quite important in China [3, 4]. At present, most regions in China have basically modernized their agriculture, and the development of rural industries has entered a phase of urban-rural industrial integration and high-quality agricultural development. The overall efficiency of China's agricultural economy is constantly improving, and market-based reforms are to blame. The level of marketization is a powerful driver of economic growth, and the diffusion effect of its externalities on the productivity of the three industries is an important force in ensuring high-quality economic growth [5]. The higher the level of marketization, the greater the evidence of market dynamism, and the higher the utilization of economic resources in a given region. Thus, it is important to investigate whether marketization can contribute to the growth of input and output efficiency in China's agriculture, which can contribute to the sound development of China's agricultural economy.

However, the rapid development of Chinese agriculture has also brought about a contradiction between environmental construction and market-oriented agricultural development. Agricultural pollution still exists because of the low utilization of agricultural resources, low penetration of technology, and other reasons, such as the high cost of agricultural inputs and the degradation of ecological production patterns. The ecological environment is the sum of all the forces or effects of the natural environment that are closely related to human life and affect human survival and development, and it is the basis for sustainable socio-economic development [6]. The agroecological environment is the collective term for the various elements that directly or indirectly affect the survival and development of agriculture, and it is an important part of the ecological environment and the material basis for agricultural economic development. In agricultural production, humans have a negative impact on the agroecological environment to a certain extent [7]. Hence, it is important to pay attention to the development of the agroecological environment at the same time as developing the agricultural economy. At the same time, the increase in income from agricultural products is closely linked to the use of fertilizer inputs, which will, in turn, lead to a considerable degree of safety risks for the quality of agricultural products [8]. The disparity in agricultural development between different regions not only affects the efficiency of agricultural production but also limits the sustainable growth of Chinese agriculture as a whole. It is evident that environmental controls have an impact on the development of the agricultural economy [9]. As a pillar of China's economic development, it is important that agriculture should adhere to a green-oriented development path.

Behind the rapid development of the agricultural economy is the deterioration of the agroecological environment and the unsustainability of agricultural development. Also, how to achieve the coordinated and sustainable development of the agricultural resources-saving, environment-friendly, and agricultural economy is the focus of research by the relevant departments [10]. Most of the existing research results are based on the agroecological perspective or the agroeconomic perspective, with both the agroecological assessment index system and the agroeconomic development index [11–13]. In addition, there are also specific measures to protect the agroecological environment and regulations and policies to develop the agricultural economy. Most of the research results on the coupling of agroecological environment and agricultural economy are based on national ecological and environmental development strategies or national agricultural development strategies [14, 15]. However, these studies do not focus on the factors influencing the agroecological environment and the actors of the agricultural economy. Even if there are studies that focus on the logical relationship between the agroecological environment and the agricultural economy, they simply assume that the agroecological environment is a condition for the development of the agricultural economy, or that the agricultural economy is an influencing factor of the agroecological environment [16]. In other words, they have failed to explore the coupling and synergy mechanisms between the two from a systemic perspective. As a result, from a systemic perspective, it is essential to develop new research perspectives and focus on the role of microlevel factors and actors in the agricultural economy, which is relevant to the discussion of agroecological environment and agricultural economy.

Agricultural ecological economic system is a compound system with specific energy conversion and material circulation rules, which is formed by the interweaving of agricultural ecological environmental system and agricultural economic system. In the agroecological economic system, people use a variety of technology and economic measures to carry out the regulation and control of the whole system, and the input of various resources makes the potential material and energy in the ecological environment resources contribute to the output of various agricultural products [17]. From the perspective of the system theory, the coupling mechanism of the agroecological economic system and agroeconomic system forms the complex relationship in the process of agroecological economic system reproduction, which is manifested as the reciprocal feedback mechanism between agricultural ecoenvironmental system and agricultural economic system [18]. The agricultural ecological environment system is the base of agricultural economic system. Agricultural economic system is the leading system of agricultural ecological environment system, and technological system is the intermediary between agricultural economic system and agricultural ecological environment system. The detailed framework of agricultural ecological economic system can be seen in Figure 2. Agroecological economic system is connected with agricultural production activities through different factors and carries out material circulation, energy flow, information exchange, and value transfer in the system [19]. Therefore, the agroecological economic system can show the characteristics of the unity of ecological environment and economy.

In fact, improving the rural living environment is of great significance to rural modernization. First of all, the construction of the rural living environment can provide a natural foundation for the construction of a beautiful countryside [20]. Because of the development of urbanization and industrialization, pollution control and resource protection are the primary objectives of rural human settlement environment construction in China. Industrial and household pollution is the main threat to the rural ecological environment, and many rural areas cannot even guarantee the basic drinking water safety [21]. The degradation of vegetation and the overexploitation of resources also put the ecosphere at risk. Over the past decade, China has made remarkable achievements in environmental protection in rural areas, which provides an ecological background for building beautiful villages. Secondly, the construction of the rural living environment can provide material basis for the construction of a beautiful countryside. Improving the rural living environment requires the construction of standardized housing, road transportation system, safe drinking water facilities, stable power supply network, drainage system, and other infrastructure [22]. These facilities are the material basis for ensuring the convenience of rural residents and living in a safe and clean environment. In addition, the construction of a rural living environment can provide the institutional foundation for the construction of a beautiful countryside [23]. To be specific, the construction of a rural living environment includes the development of democracy at the grassroots level and the creation of a fair social environment, so that the government and the people can act in accordance with laws and abide by them. It is necessary to improve the democratic supervision mechanism, protect the rights and interests of farmers, enhance their trust in the government, and make them full of hope for their future lives [24]. The perfection of the system is an important factor in the management of democracy and can provide a safe guarantee for rural residents to live and work in peace and contentment. After all, at this stage, the per capita disposable income of rural residents in China is on a steep upward trend and growing at a fast pace (Figure 3).

The GMM estimation method, which makes the orthogonal condition of the sample moment corresponding to the population moment implied by the economic model close to zero, has many advantages [25]. Firstly, the parameters of the objective function can be estimated without solving the stochastic equilibrium. Secondly, no special assumption is required for the joint distribution function of observable variables. Finally, any econometric model for which orthogonal conditions can be established can be estimated using the GMM method. The externality of instrumental variables and their correlation with endogenous variables are two very important assumptions for the use of GMM in empirical studies [26]. However, if there is only a weak correlation between the instrumental variable and the endogenous variable, a series of weak instrumental variable problems will occur. The existence of a weak instrumental variable will make the sample distribution of GMM estimation or instrumental variable estimation non-normal distribution, and the general conventional and standard statistical inference is not reliable. The weak instrumental variable problem is not a small sample problem but will also occur in large samples [27]. As a result, the subsequent development of GMM estimation in the dynamic panel model mainly follows three ideas to solve the problem of weak instrumental variables or improve their limited sample performance: improving the original instrumental variables, screening the instrumental variables in the set of instrumental variables, and using bootstrap sampling.

To sum up the realistic background, theoretical background, and policy background, the benign interaction and sustainable development of agricultural ecological environment and agricultural economy and the existing problems and research status need interdisciplinary cross-study. At the same time, it is necessary to explore the logical relationship and coupling principle between agricultural ecological environment and agricultural economy using the system view and coordination thought, to deeply analyze the target of the coordinated development of coupling system, and to take targeted policies to promote the coordinated development of an agricultural ecological environment and agricultural economy coupling system. At the same time, in view of the significant regional characteristics of agricultural ecological environment and agricultural economy, this study takes agricultural ecological environment and agricultural economy as the research object and focuses on the coordinated development of regional agricultural ecological environment and agricultural economy coupling system. What is more, marketisation is the economic driving force to improve China's agricultural production efficiency, while environmental regulation is the environmental driving force to improve its efficiency. The two complement each other and jointly promote the development of agricultural economy. On the premise of following certain environmental regulations, it will certainly have an impact on the growth of agricultural economy based on the different degrees of the market stage. Therefore, this research deeply explores the relationship between the three and discusses how market and environmental regulations directly affect agricultural production efficiency. On the basis of the traditional research, the interaction between the two is introduced, which not only enriches the research perspective but also analyzes whether the environmental regulations under the constraints of different marketization levels will affect the agricultural production efficiency of other changes.

## 2. Relationship between Environmental Regulation and Agricultural Economy

The coupled agroecological environment and agricultural economy system consists of the agroecological environment subsystem and the agricultural economy subsystem, as well as various actors. As a result, this system contains both the diversity of the agroecological environment and the diversity of the interconnectedness of the agroecological environment along with the agricultural economy. The boundaries within the coupled system and between the subsystems are more blurred, the functions are more diversified, and the system is characterized as an environmental social system.

### 2.1. Coupling System

The structure of the coupled agroecological and economic system is mainly oriented toward the interests of the actors involved in the coupled system. Through the life and production activities of the actors, the system consists of the input and output of different elements that form the material, energy, value, and information flows within the coupled system. In addition, the system can maintain a relatively stable and orderly development, thus forming the structural framework of the coupled system with the characteristics of wholeness, relevance, and hierarchy. As shown in Figure 4, the structure of the coupled system can be divided into three levels, namely the factor level, the economic and social level, and the actor level.

At the factor level, the main focus is on the form of movement and the laws of movement of the elements within the coupled system. This level can embody the primary and natural state of existence of the coupled system and is the basis and precondition for the other structural levels. At the economic and social level, the links between the elements in the system are strengthened through economic, political, cultural, and legal means. Furthermore, this level regulates the relationship between the agroecological environment and the agricultural economy, thus promoting the synergistic development of the coupled system. At the level of actors, the government, the market, and farmers are both participants in the coupled system and promoters of its harmonious development. On the one hand, it is necessary to respect the objective laws of the agroecological environment and the agricultural economy. On the other hand, it is also necessary to consider the development intentions of the actors to combine various natural, economic, and social conditions and to apply scientific and technological methods and tools to enhance the sustainability of the agroecological environment and the agricultural economy, thus promoting the synergistic development of the coupled system.

### 2.2. Objective of Developing Coupling System

The sustainable evolution of the coupled agroecological and agro economic system is fundamental to its synergistic development. In addition to this, the system is also an objective law that guides the interconnectedness and common development of all elements within the system. The goal of synergy in the coupled system is to focus on the integrated benefits of the economy, society, and the ecological environment. Without harming the agroecological environment, it is important to ensure that the economic development of agriculture meets the development needs of present and future generations. As a result, as shown in Figure 5, the objectives of the synergistic development of the coupled system are reflected in the three levels of efficiency and intensification, coordination and harmony, and the sustainable evolution of the coupled system.

At the present stage, China's agricultural economy is generally in a state of inefficient development, resulting in a low degree of intensification in the coupled system of agroecological environment and agricultural economy. The coupled system is characterized by the high input of resources, a relatively low output of agricultural products, the high consumption of agricultural production materials, and the deterioration of the ecological environment. In addition, the efficiency of agricultural production is generally lower than that of urban industries and lower than that of the agricultural economies of developed countries. To change the inefficient and sloppy development model, it is necessary to establish a scientific coupled system with ecological, economic, and social objectives and highlight the development model of high efficiency and intensification. In terms of ecological objectives, there is a need to unify direct and indirect ecological objectives to improve resilience to disasters and risks and maintain ecological security and sustainable and stable growth in ecological efficiency. In terms of economic objectives, through the positive impact of the market on the agroecological environment, a model of efficient and intensive development of the agricultural economy will be formed to promote the sustainable development of the agricultural economy. In terms of social objectives, the reform of the agricultural economic system will be deepened on the basis of the realization of ecological and economic objectives. In addition, it is necessary to establish an efficient and intensive ecological and economic development mechanism to realize the goal of efficient and intensive development of the coupled system of the agroecological environment and the agricultural economy.

### 2.3. Market Behavior Analysis

The market is the dominant force in the allocation of resources in the coupled agroecological and agroeconomic system, regulating the use of agricultural economic resources. However, because of limited rationality, externalities, and information asymmetries in the market environment, the public goods attribute of the coupled system of the agroecological environment and agricultural economy is more obvious. The coupled system is an organic link between the natural and man-made environment of agriculture, and the acquisition of agricultural outcomes is the result of the combined effect of natural resources and agricultural production. On the one hand, the production of agricultural outcomes is driven by the maximization of market interests. On the other hand, the scarcity and finiteness of natural resources inevitably require a certain limit to agricultural production, which results in the existence of a difference between private marginal costs (PMC) and social marginal costs (SMC) under market behavior, i.e., marginal external costs (MEC), as shown in Figure 6.

An important way forward for agricultural development also lies in the advancement and application of science and technology. The strategy of storing food in the land and food in technology is being implemented in depth to improve the level of security of the supply of food and other agricultural products. Firstly, it is necessary to actively enhance the level of innovation in agricultural science and technology, make full use of the resource advantage of abundant species resources, and encourage universities and research institutes to innovate, develop, and promote good crop seeds and cultivation techniques. Secondly, it is necessary to strengthen the supporting role of science and technology in agricultural development, transform scientific and technological knowledge into economic strength, enhance the technological content of agricultural products, and increase the contribution of science and technology to agricultural growth. What is more, it is necessary to vigorously promote and strengthen the status of agricultural science and technology in the development of the agricultural economy position, so that grassroots farmers can be the first to learn about the latest agricultural information.

## 3. Applications of Systematic GMM Model

### 3.1. Model Setting

In this study, dynamic panel data models are used to optimally estimate the parameters of the correlation coefficients. Dynamic GMM estimation is generally divided into two categories. In the differential GMM estimation model, the panel data advances over time and inevitably raises more instrumental variables. On the other hand, the systematic GMM model is based on differential GMM methods and can effectively overcome the endogeneity problems that arise within the model. As a result, the systematic GMM estimation method will be chosen for this research.

To further investigate the relationship between marketization, environmental regulation, and agricultural economic efficiency, it is necessary to test whether marketization and environmental regulation can directly affect agricultural economic efficiency. Therefore, the models constructed are as follows:

(1) $$\begin{array}{c} aee_{i,t}=\alpha_{0}+\alpha_{1}aee_{i,t-1}+\alpha_{2}mkt_{i,t}+\alpha_{3}er_{i,t},\\ aee_{i,t}=\alpha_{0}+\alpha_{1}aee_{i,t-1}+\alpha_{2}mkt_{i,t}+\alpha_{3}er_{i,t}+\alpha_{4}{\left(mkt^{*}er\right)}_{i,t}. \end{array}$$

Here, *aee* refers to the agricultural economic efficiency in each province, *mkt*_*i*,*t*_ refers to the marketization in each province, and *er* indicates the environmental regulation in each province.

### 3.2. Variable Selection

Given that the model in this study involves nonexpected output, it is not possible to deal with this effectively based on the SBM model. *E* is the desired optimal efficiency value, where *E* = 1 represents the strong efficiency of the decision unit. p and q represent the input and output quantities, *γ* is the radial planning parameter, and *β* is the linear combination correlation coefficient of the decision units selected for this research. Therefore, the obtaind equation is as follows:

(2) $$\begin{array}{c} E=\min\gamma -\sum_{i=1}^{p}\frac{q_{i}}{\beta_{i}}, \end{array}$$

such that

(3) $$\begin{array}{c} \left\{\begin{array}{c} \sum_{j=1}^{q}\beta_{j}+\gamma =p\\ \beta_{j}\geq 0\\ q_{i}\geq 0 \end{array}\right... \end{array}$$

Furthermore, the input of the above model can be seen in Table 1.

### 3.3. Empirical Testing

In this section, the systematic GMM model is applied to conduct the empirical testing for the related data of each province. To be specific, the results of the dynamic panel data model estimation are shown in Table 2.

The results in Table 2 show that environmental regulation and the level of marketization have a positive effect on the efficiency of the agricultural economy. Specifically, the more integrated the market environment in each region, the stronger the positive externalities of the agricultural economy. It can lead to the development of other agricultural industries in the region. At the same time, with the disappearance of market barriers, regions with backward agricultural economies can communicate with developed regions by learning new agricultural production techniques. They can continue to improve their own use of agricultural resources to increase local agricultural productivity.

The results for environmental regulation are also consistent with the findings of traditional studies. It can be concluded that the necessary environmental regulations are conducive to increased agricultural productivity. As the agricultural environment is a public good and pollution is highly external, it is no longer possible to rely solely on the internal mechanisms of the market to solve environmental pollution problems, and the inequality between inputs and outputs in the implementation process is only at the expense of greater economic costs. Therefore, strong environmental regulation is an important tool to compensate for and control these failures. By regulating the amount of agricultural resources to be used in each region to improve the efficient allocation of resources, this approach to production is ultimately closely linked to the overall development of regional agriculture.

In the model (2), the interaction term is added, and there is a negative effect of environmental regulation. It suggests that environmental regulation has a dampening effect on the efficiency of agricultural production. It argues for the importance of rational use of agricultural resources. In the initial stages of agricultural production, China's overall ecological carrying capacity is high, chemical emissions, such as pesticides, are not too polluting, and farmers consciously follow environmental regulations to ensure a high harvest for their families, which, to some extent, ensures an increase in agricultural production efficiency.

## 4. Conclusion

Based on the findings of this study, the policy recommendations that are made to improve China's agricultural economic development from the perspective of marketization and environmental regulation are as follows: firstly, the market should play a decisive role in the development of the rural economy in terms of resource allocation. Learn to rely on the power of the market to continuously promote effective linkages between agricultural production and agricultural trade in different regions of China. In addition, it is necessary to ensure that the actual factors of agricultural production in each region can be distributed and circulated on a larger scale. Also, it is necessary to eliminate the protection of local markets by local farmers, so that a large market can be established with an orderly competition of resources. It will enable regions lagging behind in agricultural development to benefit from the mutual assistance of their neighbors while giving a full play to their comparative advantages. At the same time, each region needs to formulate the necessary environmental regulations in accordance with the actual situation of the local agricultural economy, especially with regard to the regulation of agricultural production. It will ensure a steady increase in production efficiency and the full use of market and government forces to ensure quality agricultural development. However, there may be some bias and inevitably some subjectivity in this study with regard to the selection of indicators. As a result, in the future, a more in-depth empirical study can be conducted to verify the validity of the systematic GMM model, starting from the selection of indicators.

## Figures and Tables

**Figure 1:** Share of GDP by industry in China in 2021.

**Figure 2:** Framework of agricultural ecological economic system.

**Figure 3:** Per capita disposable income of rural residents in China from 2012 to 2021.

**Figure 4:** Structure of the coupled system.

**Figure 5:** Objectives of synergistic development of the coupled system.

**Figure 6:** Relationship among PMC, SMC, and MEC.

**Table 1:** Input of GMM model.

Input indictor	Factor
Labor input indicator	Number of people working in agriculture
Land input indictor	Arable land and aquaculture area
Water input indictor	Total agricultural water consumption
Energy input indictor	Total electricity consumption in agriculture

**Table 2:** Result of the dynamic panel data model estimation.

	Model (1)	Model (2)
*aee*	0.425	0.367
	0.000	0.000
*mkt*	0.025	−0.302
	0.000	0.01
*er*	1.342	1.045
	0.000	0.000
Constant	−3.389	−3.769
	0.000	0.000
*mkt* ^*∗*^ *er*		0.491
		0.000
Sargan	1	1
AR (1)	0.0074	0.0243
AR (2)	0.2013	0.318

## Data Availability

The labeled datasets used to support the findings of this study are available from the corresponding author upon request.

## References

[1] Martellozzo F., Amato F., Murgante B., Clarke K. C. (2018). Modelling the impact of urban growth on agriculture and natural land in Italy to 2030. *Applied Geography*.

[2] Lu X., Li Z., Wang H. (2022). Evaluating impact of farmland recessive morphology transition on high-quality agricultural development in China. *Land*.

[3] Cheng B., Fan C., Fu H., Huang J., Chen H., Luo X. (2022). Measuring and computing cognitive statuses of construction workers based on electroencephalogram: a critical review. *IEEE Transactions on Computational Social Systems*.

[4] Cheng B., Lu K., Li J., Chen H., Luo X., Shafique M. (2022). Comprehensive assessment of embodied environmental impacts of buildings using normalized environmental impact factors. *Journal of Cleaner Production*.

[5] Chen T., Lu H., Chen R., Wu L. (2021). The impact of marketization on sustainable economic growth-evidence from west China. *Sustainability*.

[6] Günther S., Grunert M., Müller S. (2018). Overview of recent advances in phosphorus recovery for fertilizer production. *Engineering in Life Sciences*.

[7] Wanger T. C., DeClerck F., Garibaldi L. A. (2020). Integrating agroecological production in a robust post-2020 Global Biodiversity Framework. *Nature Ecology & Evolution*.

[8] Radziemska M., Vaverková M. D., Adamcová D., Brtnický M., Mazur Z. (2019). Valorization of fish waste compost as a fertilizer for agricultural use. *Waste and Biomass Valorization*.

[9] O’Sullivan C. A., Bonnett G. D., McIntyre C. L., Hochman Z., Wasson A. P. (2019). Strategies to improve the productivity, product diversity and profitability of urban agriculture. *Agricultural Systems*.

[10] Cao Y., Zhang W., Ren J. (2020). Efficiency analysis of the input for water-saving agriculture in China. *Water*.

[11] Kiryushin V. I. (2020). Methodology for integrated assessment of agricultural land. *Eurasian Soil Science*.

[12] Duarte B., Caçador I. (2021). Iberian halophytes as agroecological solutions for degraded lands and biosaline agriculture. *Sustainability*.

[13] Dendir Z., Simane B. (2019). Livelihood vulnerability to climate variability and change in different agroecological zones of Gurage Administrative Zone, Ethiopia. *Progress in Disaster Science*.

[14] Mockshell J., Kamanda J. (2018). Beyond the agroecological and sustainable agricultural intensification debate: is blended sustainability the way forward?. *International Journal of Agricultural Sustainability*.

[15] da Costa M. B. B., Souza M., Júnior V. M., Comin J. J., Lovato P. E. (2017). Agroecology development in Brazil between 1970 and 2015. *Agroecology and Sustainable Food Systems*.

[16] Saj S., Torquebiau E., Hainzelin E., Pages J., Maraux F. (2017). The way forward: an agroecological perspective for Climate-Smart Agriculture. *Agriculture, Ecosystems and Environment*.

[17] Giraldo O. F., McCune N. (2019). Can the state take agroecology to scale? Public policy experiences in agroecological territorialization from Latin America. *Agroecology and Sustainable Food Systems*.

[18] Gallardo-López F., Hernández-Chontal M. A., Cisneros-Saguilán P., Linares-Gabriel A. (2018). Development of the concept of agroecology in Europe: a review. *Sustainability*.

[19] Chaparro-Africano A. M. (2019). Toward generating sustainability indicators for agroecological markets. *Agroecology and Sustainable Food Systems*.

[20] Brüning A., Kloas W., Preuer T., Hölker F. (2018). Influence of artificially induced light pollution on the hormone system of two common fish species, perch and roach, in a rural habitat. *Conservation Physiology*.

[21] Qu Y., Zhan L., Jiang G., Ma W., Dong X. (2021). How to Address “Population Decline and Land Expansion (PDLE)” of rural residential areas in the process of Urbanization: a comparative regional analysis of human-land interaction in Shandong Province. *Habitat International*.

[22] Ridding L. E., Watson S. C. L., Newton A. C., Rowland C. S., Bullock J. M. (2020). Ongoing, but slowing, habitat loss in a rural landscape over 85 years. *Landscape Ecology*.

[23] Thomas J. P., Jung T. S. (2019). Life in a northern town: rural villages in the boreal forest are islands of habitat for an endangered bat. *Ecosphere*.

[24] Zhou Y., Li Y., Xu C. (2020). Land consolidation and rural revitalization in China: mechanisms and paths. *Land Use Policy*.

[25] Jha C. K. (2019). Financial reforms and corruption: evidence using GMM estimation. *International Review of Economics and Finance*.

[26] Cheng S., Chen J., Liu X. (2019). GMM estimation of partially linear single-index spatial autoregressive model. *Spatial Statistics*.

[27] Andrews I., Stock J. H., Sun L. (2019). Weak instruments in instrumental variables regression: theory and practice. *Annual Review of Economics*.

